The article "The impact of newly synthesized sulfonamides on soil microbial population and respiration in rhizospheric soil of wheat (Triticum aestivum L.)" was retracted in 2022. Reasons: compromised peer review; a conflict of interest; concerns about the authorship.

# The impact of newly synthesized sulfonamides on soil microbial population and respiration in rhizospheric soil of wheat (*Triticum aestivum* L.)

**DOI:** 10.1371/journal.pone.0264476

**Published:** 2022-04-28

**Authors:** Ammara Saleem, Asma Zulfiqar, Muhammad Zeeshan Arshed, Saber Hussain, Muhammad Tajammal Khan, Marek Zivcak, Ali Tan Kee Zuan, Shrouq M. Alshahrani, Khaloud Mohammed Alarjani

**Affiliations:** 1 Molecular Plant Physiology, Institute of Botany, University of the Punjab, Lahore, Pakistan; 2 Department of Botany, Division of Science and Technology, University of Education, Lahore, Pakistan; 3 Institute of Plant and Environmental Sciences, Slovak University of Agriculture, Nitra, Slovakia; 4 Department of Land Management, Faculty of Agriculture, Universiti Putra Malaysia, UPM Serdang, Selangor, Malaysia; 5 Department of Botany and Microbiology, College of Science, King Saud University, Riyadh, Saudi Arabia; Mendel University of Agriculture and Forestry: Mendelova univerzita v Brne, CZECH REPUBLIC

## Abstract

Antibiotics released into agricultural fields through the manure of grazing animals could exert harmful impacts on soil microbes and plants. Antibiotics exert high impacts on environment than other pharmaceuticals due to their higher biological activity. However, little is known about their impacts on plants, despite indications that antibiotics exert negative effects on soil microorganisms, which ultimately harm the plants. It has been demonstrated that beneficial microorganisms promote plant growth and development under various stresses. This study evaluated the toxicity of four newly derived sulfonamides (SAs), i.e., 2-(phenylsulfonyl) hydrazine carbothioamide (TSBS-1), N, 2-bis phenyl hydrazine carbothioamide (TSBS-2), aminocarbonyl benzene sulfonamide (UBS-1), and N, N’-carbonyl dibenzene sulfonamide (UBS-2) on bacterial growth and soil microbial respiration. Each SA was tested at four different concentrations (i.e., 2.25, 2.5, 3, 4 mg/ml) against five rhizospheric bacterial strains, including AC (*Actinobacteria sp*.), RS-3a (*Bacillus sp*.), RS-7a (*Bacillus subtilis*), RS-4a (*Enterobacter sp*.), and RS-5a (*Enterobacter sp*.). Antimicrobial activity was checked by disc diffusion method, which showed that inhibition zone increased with increasing concentration of SAs. The UBS-1 resulted in the highest inhibition zone (11.47 ± 0.90 mm) against RS-4a with the highest concentration (4 mg/ml). Except TSBS-1, all sulfonamide derivatives reduced CO_2_ respiration rates in soil. Soil respiration values significantly increased till 6^th^ day; however, exposure of sulfonamide derivatives suppressed microbial respiration after 6^th^ day. On the 20^th^ day, poor respiration activity was noted at 0.23, 0.2, and 0.4 (CO_2_ mg/g dry soil) for TSBS-1, UBS-1, and UBS-2, respectively. Our results demonstrate that sulfonamides, even in small concentrations, significantly affect soil microbial population and respiration. Soil microbial respiration changes mediated by sulfonamides were dependent on length of exposure and concentration. It is recommended that antibiotics should be carefully watched and their impact on plant growth should be tested in the future studies.

The article "The impact of newly synthesized sulfonamides on soil microbial population and respiration in rhizospheric soil of wheat (Triticum aestivum L.)" was retracted in 2022. Reasons: compromised peer review; a conflict of interest; concerns about the authorship.

## Introduction

Antibiotics exert varying impacts on bacteria, algae, and other microbes. Initially, any agent with biological activity against living organisms was regarded as an antibiotic. However, now it exclusively refers to the compounds that have antibacterial, antifungal, or antiparasitic properties [1]. The use of various antibiotics on humans and animals can lead to environmental pollution. Antibiotic metabolites have been found in soil, manures, sediments, industrial waste, groundwater, surface water, and drinking water [2, 3]. When animal dung containing excreted antibiotics is used as plant food, these chemicals are released into the environment [4]. Sulfonamide is widely used in livestock farming and has been used to treat a variety of bacterial diseases. Due to poor management, they are excreted into the soil after treatments and these are extremely hazardous [5].

Unlikely, pesticides on farming land and antibiotics are not getting much consideration as environmental pollutants yet [6]. Different antibiotics are exposed to the environment in very different ways [7]. Sulfonamides may impair the growth of plants, leaves, and roots at concentrations of several hundred mg/L [8].

Antibiotic residues pose negative impacts to microbial processes in the environment [9]. Antibiotic output continues to increase, with total annual use rising from 100,000 to 200,000 tones globally [10]. India, China, and Pakistan are the top antibiotic consumers among poor and middle-income countries of the world [11]. Fluoroquinolones and sulfonamides are two antibiotic families found in high amounts in feces [12, 13].

Wheat (*Triticum aestivum* L.) is one of the world’s most important food crops [14], grown worldwide in several cropping regions [15]. The global wheat production during 2020–2021 was over 768.9 million metric tons [16]. Future predictions suggest that there will be an increased demand for wheat (by 60% of the current production) till 2050 to feed an estimated 9.7 billion population in the world. Therefore, global importance of wheat is the best justification for conducting research on rhizospheric microbiome recognition and their activity in the rhizospheric soil of wheat cultivars [9]. The rhizosphere of wheat plants is highly diverse and thirty OTUs has been detected, including *Alphaproteobacteria*, *Betaproteobacteria*, *Deltaproteobacteria*, *Gammaproteobacteria*, *Actinobacteria*, *Bacilli*, *Clostridia*, and uncultivable bacteria [17]. The global importance of wheat necessitates the recognition of rhizospheric microbiome of the most popular wheat cultivars. The selection of best-quality cultivars is a key element as it creates a possibility of cultivation of high-quality wheat varieties in a specific field and climatic zone [18].

The article "The impact of newly synthesized sulfonamides on soil microbial population and respiration in rhizospheric soil of wheat (Triticum aestivum L.)" was retracted in 2022. Reasons: compromised peer review; a conflict of interest; concerns about the authorship.

Maintaining a high crop yield is crucial for profit and food supply for global population. Plant growth-promoting organisms have attracted significant interest recently because of their potential to help plants growth under adverse conditions. Plant growth-promoting organisms use a variety of processes to promote root growth and development. These organisms in the rhizosphere can assist plants in reducing stress and improving growth and development [19]. Recently, there has been increased interest in beneficial rhizobacterium associated with cereal crops, and several studies have clearly demonstrated the positive and beneficial effects of plant growth promoting rhizobacteria (PGPR) on growth and yield of various crops, especially wheat [20]. Several beneficial free-living rhizobacteria have been termed as PGPR, including, but not limited to *Acinetobacter*, *Acetobacter*, *Alcaligenes*, *Arthrobacter*, *Azotobacter*, *Azospirillum*, *Bacillus*, *Burkholderia*, *Beijerinckia*, *Enterobacter*, *Flavobacterium*, *Methylobacterium*, *Pseudomonas*, *Rhizobium*, *Paenibacillus* and *Pantoea* [21].

Accumulations of different antibiotics, including sulfonamides harmed the function and activity of microorganism and reduce soil enzymatic activity. Antibiotics in soil can bring constant changes in organisms and plants and exert harmful impacts on soil microbes and their functions which are important for decomposition and nutrient cycling. Antibiotic residues are considered among one of those factors which have adverse effects on the microbial processes in the environment [22]. Antibiotic accumulations, especially sulfonamides, harm microorganism function and activity and diminish soil enzymatic activity. Antibiotics contained in soil can cause organisms and plants to undergo continuous modifications and this could harm soil bacteria and their functions, which are critical for decomposition and nutrient cycling [23]. Sulfonamides delay the assembly of dihydropteroate of folic acid, which reduces bacterial reproduction [24]. Antibiotics may potentially have an impact on the diversity of soil microorganisms [25], soil microbial action [26], enzyme activity [27], and carbon and nitrogen cycling [28]. The impacts of sulfonamides on the functional, structural, and genetic diversity of soil microorganisms have been reported in earlier study [29]. Previous research has shown that most of the antibiotics released into the agricultural environment come from the direct application of organic manure, which affects microbial communities.

The article "The impact of newly synthesized sulfonamides on soil microbial population and respiration in rhizospheric soil of wheat (Triticum aestivum L.)" was retracted in 2022. Reasons: compromised peer review; a conflict of interest; concerns about the authorship.

Abiotic and biotic stressors can change plant-pest interactions by increasing the susceptibility of plants to pathogenic microbes and insects [30], which interfere with the action of plant growth-promoting rhizospheric bacteria essential for plant growth and as well as suppress the diseases [31]. This study was conducted to infer impact of four newly synthesized sulfonamides on isolated native strains from rhizosphere of wheat cultivar ‘Chakwal-50’. Furthermore, present research focused on the susceptibility of soil microbes and microbial respiration in the rhizospheric soil of wheat.

## Materials and methods

### Experimental site

The current study was conducted at Botanical Garden, University of the Punjab, Lahore, Pakistan (31°30′7.35′′N and 74° 16′57.35′′E latitude and longitude). The physical and chemical properties of soil were analyzed before the experiment. Soil analysis revealed that the experiment soil had 5.9 pH, EC was 1.9 dS m^-1^, organic matter content was 0.89%, available nitrogen was 0.2%, available potassium was 139 mg/kg, available phosphorus was 2.5 mg/kg and saturation was 44%. The soil had loamy texture.

### Sample collection

The four new sulfonamide derivatives, i.e., 2-(phenylsulfonyl) hydrazinecarbothioamide (TSBS-1), N, 2 bis (phenylhydrazine) carbothioamide (TSBS-2), (aminocarbonyl) benzene sulfonamide (UBS-1) and N, N’ carbonyldibenzenesulfonamide (UBS-2) were obtained from School of Chemistry, University of Punjab, Lahore, Pakistan.

Soil samples were collected from the rhizospheric area of wheat (*Triticum aestivum* L.) variety ‘Chakwal-50’ for isolation of bacteria. Five isolated bacterial strains, i.e., AC (*Actinobacter spp)*, RS-3a (*Bacillus spp*.), RS-7a (*Bacillus subtilis*), RS-4a (*Enterobacter spp*.) and RS-5a (*Enterobacter spp*.) isolated from the wheat rhizosphere were included in the study. These strains belonged to Microbiology laboratory, Institute on Botany, University of the Punjab, Lahore, Pakistan. Strains were kept at 80 °C and revived in nutrient broth at 30 °C for 48 hours.

Bacterial suspensions were prepared as per McFarland’s standard. One-day-old bacterial cultures were used for the preparation of inoculums and maintained at 1.5 × 10^8^ [32]. Four dilutions, i.e., 2.25, 2.5, 3, and 4 mg/ml of each sulfonamide derivatives were prepared in DMSO for antibacterial essay and soil microbial respiration test. The experiment was laid out according to completely randomized design (CRD) with three replicates. Five bacterial strains were tested against different sulfonamides and their 4 different doses.

The article "The impact of newly synthesized sulfonamides on soil microbial population and respiration in rhizospheric soil of wheat (Triticum aestivum L.)" was retracted in 2022. Reasons: compromised peer review; a conflict of interest; concerns about the authorship.

### Antibacterial assay

The antibacterial assay was done by disc diffusion method by using four different concentrations (2.25, 2.5, 3, and 4 mg/ml) against all bacterial strains. Ciprofloxacin used as a standard drug was regarded as positive control, while DMSO (dimethyl sulfoxide) as negative control [33]. In disc diffusion method, agar plants were inoculated with standardized inoculum by spreading 100 *μ*L of bacterial suspensions onto Petri plates. After the dilution’s preparation, 5 *μ*L of desired dilution of antibiotic was loaded on 6 mm filter paper disc individually. Afterwards, Petri plates were inverted to prevent moisture, and incubated at 37 °C for 24 hours. All the tests were repeated four times. The antibacterial action was detected after incubation and assessed as inhibition zone with transparent ruler from back of the plate [34].

### Soil respiration test

Fifty (50) grams of soil samples were put in plastic cups and loaded with each sulfonamide solution, separately. Further, 1 mL of 0.1 M glucose solution and 10 mL of distilled water were also added to maintain the soil moisture at 25%. The test soil was kept overnight. Another cup was filled with 20 mL of 0.15 N NaOH. These plastic cups with test soil and sodium hydroxide were placed in an air-tight jar and incubated at 25 °C in darkness. The control had a blank plastic cup without soil but 20 mL of 0.15 N NaOH. The soil respiration value (CO_2_) was calculated by titration of NaOH present in the bottommost of each jar with 0.1 N HCl. The titration was done after different days of interval (3, 6, 9, 12, 16, and 20 days). Each treatment has four replicates.

The value of soil respiration was determined by the formula according to Yao et al. [35].


$$\text{Respiration}\;\text{value}\;\left(\text{mg}\;{\text{CO}}_{2}\;{\text{g}}^{-1}\;\text{dry}\;\text{soil}\right)=\text{Blank-titer}/0.1/44/50$$

### Statistical analysis

The data obtained for different characters were tested for normality which indicated that data had a normal distribution. Two-way analysis of variance was used to test the significance in the data. Duncan’s multiple range post-hoc test was used to observe the differences (p≤0.05) among means where ANOVA indicated significant differences. All statistical analysis were carried out on SPSS statistical software.

The article "The impact of newly synthesized sulfonamides on soil microbial population and respiration in rhizospheric soil of wheat (Triticum aestivum L.)" was retracted in 2022. Reasons: compromised peer review; a conflict of interest; concerns about the authorship.

## Results

### Antibacterial assay

Results for antibacterial assay of all sulfonamide derivatives show that all antibiotics exerted negative impact on rhizospheric bacteria (Table 1). All sulfonamide derivatives exhibited antibacterial activity against tested bacterial strains, except for TSBS-1, which has no antibacterial activity against RS-7a at the lowest concentration (2.25 mg/ml). The results of all treatments were compared with ciprofloxacin, a standard antibiotic, as a positive control and dimethyl sulfoxide (DMSO), a negative control. The DMSO had no antibacterial activity.

**Table 1:** Antibacterial activity of newly derived sulfonamides by disc diffusion method against five different rhizospheric bacteria.

Sulfonamides	Concentration	Bacterial strains diameter of zone of inhibition (mm ± SD)				
	(mg/ml)	AC	RS-3a	RS-7a	RS-4a	RS-5a
**TSBS-1**	2.25	6.33 ± 0.57	6.58 ± 1.52	0	6.65 ± 0.73	6.16 ± 0.53
	2.5	7.81 ± 0.96	7.64 ±0.77	6.81 ± 0.83	7.75 ± 0.78	7.46 ± 0.64
	3	8.75 ± 0.41	8.44 ± 0.36	7.46 ± 0.50	8.55 ± 0.30	8.29 ± 0.36
	4	10.59 ±0.62	9.94 ± 0.07	8.83 ± 0.76	10.07 ± 0.64	9.57 ± 0.27
**TSBS-2**	2.25	6.07 ± 0.87	6.24 ± 0.32	5.43 ± 0.49	6.30 ± 0.519	6.21 ± 0.92
	2.5	7.151 ±1.03	7.11 ± 1.08	6.81 ± 0.83	7.75 ± 0.78	7.67 ± 0.74
	3	8.41 ± 1.51	8.70 ± 0.41	8.74 ± 1.09	9.07 ± 0.88	8.64 ± 0.62
	4	10.66 ±1.16	9.89 ± 0.67	9.46 ± 1.23	10.64 ± 0.24	9.99 ± 0.97
**UBS-1**	2.25	6.78 ± 1.06	6.33 ± 0.93	5.65 ± 1.13	6.48 ± 0.40	6.66 ± 0.41
	2.5	7.49 ± 0.48	7.69 ± 1.09	6.99 ± 0.94	7.36 ± 0.52	7.70 ± 1.12
	3	8.95 ± 1.35	8.11 ± 0.75	8.66 ± 0.57	9.4 ± 0.25	9.12 ± 0.27
	4	11.29 ±1.16	10.91 ± 0.92	10.66 ± 1.16	11.47 ± 0.90	11.01 ± 1.62
**UBS-2**	2.25	7.07 ± 0.53	7.12 ± 0.45	6.23 ± 0.49	7.35 ± 0.92	6.95 ± 1.91
	2.5	8.01 ± 1.21	7.67 ± 2.07	7.37 ± 0.45	8.16 ± 1.60	8.04 ± 1.40
	3	9.32 ± 1.42	8.77 ± 1.06	8.66 ± 0.32	8.89 ± 0.18	8.89 ± 1.01
	4	10.99 ±1.01	10.66 ± 0.58	10.78 ± 0.45	10.92 ± 1.83	11.05 ± 1.23
**Ciprofloxacin**	4	9.97 ± 1.11	9.43 ± 0.68	10.01 ± 1.26	9.91 ± 1.66	10.03 ± 1.02
**DMSO**	4	-	-	-	-	-

TSBS-1 {2-(phenylsulfonyl) hydrazine carbothioamide}, TSBS-2 {N,2-bis phenyl hydrazine carbothioamide}, UBS-1 {(aminocarbonyl) benzene sulfonamide}, UBS-2 {N,N’ (carbonyl) dibenzene sulfonamide}, AC (*Actinobacteria* sp.), RS-3a (*Bacillus* sp), RS-7a (*Bacillus subtilis*), RS-4a (*Enterobacter* sp.) and RS-5a (*Enterobacter* sp.), DMSO (Dimethyl sulfoxide) values are in mean ± SD.

In comparison of all sulfonamide derivatives UBS-1 exhibited the highest inhibition zone (11.47 ± 0.90 mm) against RS-4a at the highest concentration (4 mg/ml). Furthermore, all other strains, including AC, RS-3a, RS-7a, and RS-5a found susceptible to UBS-1 with inhibition zones of 11.29 ± 1.16, 10.91 ± 0.92, 10.66 ± 1.16, and 11.01 ± 1.62, respectively.

The article "The impact of newly synthesized sulfonamides on soil microbial population and respiration in rhizospheric soil of wheat (Triticum aestivum L.)" was retracted in 2022. Reasons: compromised peer review; a conflict of interest; concerns about the authorship.

However, UBS-2 has greater antibacterial potential against RS-7a and RS-5a with inhibition zone of 10.01 ± 1.26 and 10.03 ± 1.02, respectively at 4 mg/ml concentration. The zone of inhibition in both tested bacterial strains was significantly higher with respect to other strains and sulfonamide derivatives.

### Soil microbial respiration (CO_2_ mg/g dry soil)

All sulfonamides had negative effect on soil microbial respiration. The results of this study revealed that sulfonamide derivatives inhibit microbial respiration which was time and concentration dependent. Soil respiration values increased significantly till 6^th^ day; however, 6^th^ day after exposure to sulfonamide derivatives, soil respiration decreased significantly (p<0.05).

The effective concentration in the first 3 days was calculated as 4 mg/ml for UBS-1 with an average value of 1.6 (CO_2_ mg/g dry soil), while little effects were observed at other concentrations (Fig 1). Within 4–6 days, each sulfonamide derivative showed significant increases in soil respiration activity, but substantial differences were only seen at the higher concentrations. On the other hand, soil microbial respiration dropped dramatically on days 7–9, but a considerable decrease was recorded for the TSBS-1 value of 0.67 (CO_2_ mg/g dry soil).

**Fig 1:** Alteration in microbial respiration in the soil due to UBS-1 exposure at different incubation durations (3, 6, 9, 12, 16 and 20 days), n = 4, vertical bars represent means ± standard errors of means. Means sharing different letters are statistically significant (p <0.05).

When compared to other incubation periods, the inhibition rates were quite variable on days 10–12 and 13–16; however, there was no significant difference between 12^th^ and 16^th^ day at each concentration level. However, at a high concentration level (4 mg/ml), the results were substantial for UBS-1, with a 0.5 inhibition rate on day 12 (Fig 1) and a 0.4 inhibition rate for UBS-2 on day 16 (Fig 2).

**Fig 2:** Alteration in microbial respiration in the soil due to UBS-2 exposure at different incubation durations (3, 6, 9, 12, 16 and 20 days), n = 4, vertical bars represent means ± standard errors of means. Means sharing different letters are statistically significant (p <0.05).

In contrast to the activities in the first few days, a major decrease in respiration activity was observed in later incubation periods. Soil respiration activity was markedly hindered towards the end of incubation period even at small concentrations. Microbial respiration activity diminished as the concentration of each treatment and time of exposure increased.

The article "The impact of newly synthesized sulfonamides on soil microbial population and respiration in rhizospheric soil of wheat (Triticum aestivum L.)" was retracted in 2022. Reasons: compromised peer review; a conflict of interest; concerns about the authorship.

Based on the concentrations (4 mg/ml) and time (20 days), poor respiration activity was noted at 0.23, 0.2, and 0.4 (CO_2_ mg/g dry soil) for TSBS-1, UBS-1, and UBS-2, respectively (Figs 1–3). The results of TSBS-2 at 3 mg/ml were more significant than 4 mg/ml, with mean values of 0.29 (CO_2_ mg/g dry soil) and 0.4 (CO_2_ mg/g dry soil), respectively (Fig 4).

**Fig 3:** Alteration in microbial respiration in the soil due to TSBS-1 exposure at different incubation durations (3, 6, 9, 12, 16 and 20 days), n = 4, vertical bars represent means ± standard errors of means. Means sharing different letters are statistically significant (p <0.05).

**Fig 4:** Alteration in microbial respiration in the soil due to TSBS-2 exposure at different incubation durations (3, 6, 9, 12, 16 and 20 days), n = 4, vertical bars represent means ± standard errors of means. Means sharing different letters are statistically significant (p <0.05).

## Discussion

In this study we focused on four novel synthetic sulfonamides, i.e., TSBS-1 {2-(phenylsulfonyl) hydrazine carbothioamide}, TSBS-2 {N,2-bis phenylhydrazine carbothioamide}, UBS-1 {(aminocarbonyl) benzene sulfonamide}, and UBS-2 {N,N’ (carbonyl) dibenzene sulfonamide}.

Table 1 reveals that all sulfonamide derivatives have negative effect on soil microbes with statistically significant differences. Previous literature also indicated that Gram-negative and Gram-positive bacteria are susceptible to sulfonamides. They are synthetic antimicrobials with the ability to impede the microbe’s folic acid pathway [36].

All synthesized sulfonamides inhibited the growth of isolated bacterial strains even at low concentration (2.25 mg/ml) except for TSBS-1 against RS-7a and did not show any inhibition zone at 2.25 mg/ml. However, all other bacteria were found susceptible to TSBS-1. Sulfonamides are a synthetic drug with a wide range of activity against all positive and negative bacteria, protozoa, and toxoplasma [37]. Sulfonamides exert their effect by targeting dihydropteroate synthase (DHPS) enzyme, which catalyzes the folic acid pathway in bacteria and results in the stoppage of folate biosynthesis in microorganism cells; thus, restraining microorganism growth [38].

Soil respiration measured as cumulative CO_2_ decreased significantly with increasing concentrations of sulfonamide for up to 3 days only (Figs 1–4). Soil respiration significantly decreased with increasing concentrations of sulfamethoxazole and trimethoprim in the soil [39]. The earlier study also discovered that antibiotic sulfadiazine inhibited microbial activity in manure for up to 4 days after application, and that the effective doses for sulfamethoxazole in the first 2 days were calculated to be 7 mg/kg. Antibiotics may potentially have an impact on the diversity of soil microorganisms [25], soil microbial action [26], enzyme activity [27].

The article "The impact of newly synthesized sulfonamides on soil microbial population and respiration in rhizospheric soil of wheat (Triticum aestivum L.)" was retracted in 2022. Reasons: compromised peer review; a conflict of interest; concerns about the authorship.

Until the 6^th^ day, the levels of soil respiration greatly increased. Previous research has also found an increase in soil respiratory activity [40]. Each sulfonamide derivative demonstrated statistically significant increases in soil respiration activity within 4–6 days in our investigation. Our findings are consistent with Thiele-Bruhn et al. [41]. According to Thiele-Bruhn et al. [41], increasing soil respiration is linked to a decrease in the amount of antibiotics that are available, as well as increased microorganism adaption and resistance. The impacts of sulfonamides on the functional, structural, and genetic diversity of soil microorganisms have also been reported [29].

After 6^th^ day exposure of sulfonamide derivatives to the soil (9, 12, 16, 20 day), the soil respiration decreased significantly (p<0.05). Soil respiration activity was markedly hindered towards the end of the day even at small concentrations. In comparison to antibiotic concentrations (up to 91 mg/kg) in manure and soils [42], inhibitory effects from antibiotics such sulfonamides in the environment are more expected. Soil respiration activity is important for higher production of wheat. Several abiotic stresses are already affecting the productivity of different crops including wheat [43–47]. Therefore, antibiotics should be carefully monitored and their impact on plant growth should be quantified in the future studies.

## Conclusions

The varied terrestrial toxicological effects of sulfonamide antibiotics were investigated using several bioassays, including antibacterial essay and soil respiration. In conclusion, (aminocarbonyl) benzene sulfonamide (UBS-1) exhibited highest zone of inhibition against all tested bacterial strains. Soil respiration activity was markedly hindered towards the end of the incubation period even at small concentrations of TSBS-1 {2-(phenylsulfonyl) hydrazine carbothioamide}, TSBS-2 {N, 2-bis phenyl hydrazine carbothioamide}, UBS-1 {(aminocarbonyl) benzene sulfonamide}, and UBS-2 {N,N’ (carbonyl) dibenzene sulfonamide}. The results of this study can be applied to the environmental risk assessment of sulfonamide, including estimation of the determination of sulfonamide in the environment. Sulfonamides have a negative influence on the soil microbiome, and some soil microorganisms that are unable to resist such stressors, so it is difficult to retain soil fertility and plant development as well. Soil microbial respiration changes mediated by sulfonamides were dependent on length of exposure and concentration. It is recommended that antibiotics should be carefully watched and their impact on plant growth should be tested in the future studies.
